The article "Understanding How Patients With Lumbar Radiculopathy Make Sense of and Cope With Their Symptoms" was retracted in 2025. Reasons: lack of ethics approval or compliance; concerns about the citations; concerns about the welfare of human subjects.

# Understanding How Patients With Lumbar Radiculopathy Make Sense of and Cope With Their Symptoms

**DOI:** 10.7759/cureus.56987

**Published:** 2024-03-26

**Authors:** Pooja Samant, Poonam Tawde, Divya N Tawde

**Affiliations:** 1 Physical Therapy, Cardiff University, Cardiff, GBR; 2 Medicine, Avalon University School of Medicine, Willemstad, CUW; 3 Medicine, Chandler Regional Medical Center, Chandler, USA; 4 Health Sciences, D&D Global Co, Toronto, CAN

**Keywords:** qualitative evidence synthesis, common sense model of self-regulation (csm), self-management, coping strategies, illness representation, lumbar radiculopathy

## Abstract

Lumbar radiculopathy, characterized by pain radiating along a nerve root, significantly diminishes the quality of life due to its neuropathic nature. Patients' understanding of their illness and the coping strategies they employ directly influence how they manage their condition. Understanding these illness representations from the patient's perspective is crucial for healthcare providers seeking to optimize treatment outcomes. This study adopted a qualitative interpretive/constructive paradigm to explore this dynamic. A qualitative evidence synthesis approach, utilizing best-fit framework synthesis for data extraction, was applied to analyze primary qualitative studies focused on patient experiences with lumbar radiculopathy. Using SPiDER (Sample, Phenomenon of interest, Design, Evaluation, Research type) to guide the search strategy, extracted data was mapped against the Common-Sense Model of Self-Regulation (CSM) framework. Sixteen studies, with moderate to minor methodological quality concerns, were included in the analysis. Data mapping across CSM domains generated 14 key review findings. Results suggest that patients with high-threat illness representations often exhibit maladaptive coping behaviors (e.g., activity avoidance) driven by emotional responses. In contrast, problem-solving techniques appear to contribute to positive outcomes (e.g., exercise adherence and effective self-management) in patients who perceive their condition as less threatening. These findings highlight the potential benefits of interventions designed to reduce perceived threat levels and enhance self-efficacy in patients with lumbar radiculopathy, leading to improved self-management and ultimately better health outcomes.

## Introduction and background

Neuropathic pain, mainly characterized by prickling, burning, or electric shock-like sensations, presents a formidable challenge, often resisting treatment and leading to poor post-therapy outcomes and diminished patient satisfaction. It typically manifests as a chronic and severe condition, significantly impacting an individual's biopsychosocial and economic well-being and consequently lowering their quality of life [1-3]. A systematic review was conducted to assess the epidemiology of neuropathic pain and its repercussions on life quality. This analysis revealed a prevalence of diminished quality of life, heightened economic and psychological (anxiety/depression) burdens, and overall reduced health across physical, psychological, and social dimensions in patients with neuropathic pain compared to those without such characteristics. Thus, it confirms the deleterious effects of neuropathic pain on various aspects of life, often arising from lesions or diseases of the somatosensory system. Lumbar or lumbosacral radiculopathy emerges as the most prevalent type of neuropathic pain [3].

The article "Understanding How Patients With Lumbar Radiculopathy Make Sense of and Cope With Their Symptoms" was retracted in 2025. Reasons: lack of ethics approval or compliance; concerns about the citations; concerns about the welfare of human subjects.

Reviews aiming to delineate low back pain and its neuropathic variations identify radiculopathy as a neurological condition characterized by a sensory or motor conduction block. While sensory conduction block presents as dermatomal numbness, motor conduction block manifests as myotomal weakness, without necessarily involving pain. Radiculopathy may or may not coincide with pain. Conversely, radicular pain results from ectopic discharge originating from a dorsal root or ganglion, commonly attributed to intervertebral disc prolapse and inflammation of affected nerve roots. It typically presents as an electric, lancinating, or shock-like sensation along the lower extremity, driven by heterospecific discharge in the involved nerve rather than exclusive nociceptive afferents. Both radiculopathy and radicular pain can occur concurrently or independently, with lumbar or lumbosacral radiculopathy being the focal point of this study [4].

Symptoms of neuropathic pain encompass continuous or paroxysmal spontaneous pain, dysesthesia, allodynia, and hyperalgesia. Spontaneous pain arises from ion channel modulation at nerve damage sites, independent of external stimuli. Evoked pain, stimulus-dependent, includes allodynia, triggered by non-noxious stimuli, and hyperalgesia, an exaggerated response to normally painful stimuli. Repeated spontaneous and evoked pain, stemming from diminished descending pain control or heightened neuro-immune responses, can perpetuate neuropathic pain [5,6].

Lumbar radiculopathy, being neuropathic, significantly impairs biopsychosocial functioning compared to nociceptive low back pain or other musculoskeletal conditions. Patients with lumbar radiculopathy exhibit higher pain severity and functional disability scores, hindering daily activities and work productivity and leading to increased healthcare utilization and economic burden. These psychological stressors activate the hypothalamus-pituitary-adrenal axis, exacerbating sympathetic activity and cortisol levels and further complicating the physical, psychological, and socioeconomic aspects of patients' lives [7,8].

The article "Understanding How Patients With Lumbar Radiculopathy Make Sense of and Cope With Their Symptoms" was retracted in 2025. Reasons: lack of ethics approval or compliance; concerns about the citations; concerns about the welfare of human subjects.

Physiotherapy interventions aim to restore self-management and functional capacity while addressing patients' beliefs about their condition through a cognitive-behavioral approach. Functional restoration programs, combining functional exercises and cognitive restructuring, have shown significant improvements in disability outcomes and work status, particularly in patients with long-term symptoms and poor prognostic indicators. Conservative treatments targeting key factors in initiating and perpetuating lumbar radiculopathy symptoms, including manual therapy and cognitive-behavioral techniques, demonstrate sustained improvements in disability outcomes [9-11].

Systematic reviews of clinical guidelines advocate for educational interventions and physical activity as cornerstone treatments for lumbar radiculopathy. However, successful treatment implementation hinges on patients' perceptions of their condition and response to pain, emphasizing the importance of addressing their beliefs [12,13]. The common-sense model elucidates how patients' illness representations influence treatment-seeking behaviors and adherence. Physiotherapists, by understanding patients' illness and treatment representations, can tailor interventions to enhance self-management and treatment outcomes, emphasizing the critical role of patient motivation in behavior change [14,15].

## Review

This research is grounded in the interpretive/constructive paradigm, which subscribes to a relativist ontology, suggesting that reality is not singular but rather multifaceted, and a subjective epistemology, which asserts that reality is socially constructed through individuals' cognitive processes [16]. Central to this paradigm is the concept of sense-making, which emphasizes the significance of the meaning attributed to experiences. It allows researchers to delve into and comprehend the diverse realities constructed through interactions with subjects [17,18]. Qualitative methods are predominantly employed by researchers to embrace this interpretive paradigm, enabling them to move beyond numerical data and explore human narratives about their thoughts. Consequently, this approach yields richer descriptions of phenomena and enhances understanding of human expressions and perspectives [19,20]. Thus, qualitative approaches are instrumental for health practitioners in probing patients' experiences to grasp the intricate cognitive and affective factors influencing these experiences [21,22]. Consequently, the synthesis of knowledge provided by qualitative investigations analyzing human experience is imperative for therapists to make evidence-based decisions when confronting the unpredictable nature of lumbar radiculopathy pain [23,24].

The article "Understanding How Patients With Lumbar Radiculopathy Make Sense of and Cope With Their Symptoms" was retracted in 2025. Reasons: lack of ethics approval or compliance; concerns about the citations; concerns about the welfare of human subjects.

Qualitative evidence synthesis (QES) is a systematic review form that synthesizes the findings of primary qualitative studies in a systematic manner [25]. The outcomes of a QES can offer insightful interpretations of a condition's impact as well as a deeper understanding of patients' experiences, opinions, beliefs, and treatment goals [26-28]. Hence, this study employed QES in line with the constructivist paradigm to underpin the understanding and interpretations of how patients make sense of their experiences with lumbar radiculopathy symptoms. This involves forming meaning from these interpretations to comprehend the cognitive, affective, and behavioral responses derived through this sense-making process [29]. The Preferred Reporting Items for Systematic Reviews and Meta-Analyses (PRISMA) guidelines were utilized to conduct and report the study (see Appendix 1) as they facilitate transparent, comprehensive, and accurate documentation of methods to identify, select, appraise, and synthesize primary studies and study results, along with the rationale behind them [30].

Study selection

Data and Information Sources

Following the formulation of the question, sampling, the subsequent step, was carried out by searching various computerized databases accessed from the learning center [31]. These included the Cumulative Index of Nursing and Allied Health Literature (CINHAL)/Medical Literature Analysis and Retrieval System Online (MEDLINE)/PubMed for a broad array of medical and healthcare-related literature from diverse disciplines. The Cochrane Handbook and the Joanna Briggs Institute recommend MEDLINE CINHAL, supplemented by PsychINFO for additional content-specific searches. The ProQuest database was consulted for literature pertinent to health social science and psychology related to the topic. Further studies were identified by scrutinizing the reference lists and citing articles of significant papers.

Search Strategy

The literature search employed search terms derived from key concepts and their synonyms, following the SPiDER framework (Table 1). This framework's terminologies are tailored for qualitative research components, facilitating efficient scanning of search results [32]. Search terms were crafted by amalgamating free texts with corresponding database headings and subheadings, and searched within titles, abstracts, or keywords. Key concepts encompassed lumbar radiculopathy, experiences and beliefs, interviews/focus groups, and qualitative research. To broaden the search scope, these terms were expanded using truncations and combined using Boolean operators AND (same criteria) OR (between criteria). An illustrative example of this comprehensive strategy is detailed in Table 2.

The article "Understanding How Patients With Lumbar Radiculopathy Make Sense of and Cope With Their Symptoms" was retracted in 2025. Reasons: lack of ethics approval or compliance; concerns about the citations; concerns about the welfare of human subjects.

**Table 1:** SPiDER concepts Source: Ref. [32]. SPiDER: Sample, Phenomenon of interest, Design, Evaluation, Research type.

Sample	Phenomenon of interest	Design	Evaluation	Research type
Sciatica, lumbar radiculopathy	Making sense	Interview, focus, groups, case study	Patient experiences	Qualitative research

**Table 2:** Search strategy (using key concepts)

#	Search strategy
1	(MM "Radiculopathy")
2	(MM "Sciatica")
3	(MM "Sciatic Neuropathy")
4	(MM "Intervertebral Disc Displacement")
5	(MM "Lumbosacral Region")
6	(MM "Nerve Compression Syndromes")
7	1 OR 2 OR 3 OR 4 OR 5 OR 6
8	((disc or discs or disk or disks) and (displacement or hernia* or protru* or avulsion*)) AB, TI, TX
9	((nerve root or nerve roots) and (compress* or entrap* or inflammat* or disorder*)) AB, TI, TX
10	sciatic* AB, TI, TX
11	radicular or radicular pain or leg pain AB, TI, TX
12	sciatica AB, TI, TX
13	lumbar radiculopathy AB, TI, TX
14	8 OR 9 OR 10 OR 11 OR 12 OR 13
15	7 OR 14
16	Interview AB, TX
17	Focus Groups AB, TX
18	Case Study AB, TX
19	Open-ended questions AB, TX
20	16 OR 17 OR 18 OR 19
21	Experience* AB, TI, TX
22	View* AB, TI, TX
23	Opinion* AB, TI, TX
24	Attitude* AB, TI, TX
25	Perce* AB, TI, TX
26	Belie* AB, TI, TX
27	Feel* AB, TI, TX
28	Know* AB, TI, TX
29	Understand* AB, TI, TX
30	Sense
31	Meaning
32	21 OR 22 OR 23 OR 24 OR 25 OR 26 OR 27 OR 28 OR 29 OR 29 OR 30 OR 31
33	(MM "Qualitative Research+")
34	qualitative study AB, TI, TX
35	qualitative methods AB, TI, TX
36	15 AND 20 AND 30 AND 32 AND 35

Eligibility

Inclusion Criteria

Primary studies utilizing both qualitative methods of data collection (interviews and focus groups with open-ended questions) and qualitative methods of data analysis (framework synthesis, grounded theory, and thematic analysis) were considered for inclusion in this study [33]. Articles interpreting the experiences of individuals afflicted with lumbar radiculopathy, with or without radicular pain, were included [34-36]. Articles published between January 2005 and June 2022 were eligible. This timeframe of the past 15 years was chosen to align with the proliferation of various treatments, including spinal injections, physiotherapy, surgical procedures, pharmacological treatments, and changes in pain neuroscience education delivery. Thus, it aims to assess patients' experiences in correspondence with treatment advancements and information dissemination. Peer-reviewed articles were included. Eligibility screening involved two stages: initial screening based on title and abstract, followed by full-text screening, with articles excluded accordingly.

The article "Understanding How Patients With Lumbar Radiculopathy Make Sense of and Cope With Their Symptoms" was retracted in 2025. Reasons: lack of ethics approval or compliance; concerns about the citations; concerns about the welfare of human subjects.

Exclusion Criteria

Studies employing qualitative methods for data collection but not employing qualitative analysis methods for data analysis were excluded. Non-English articles (due to limited translation resources) and gray literature were excluded, despite potential language bias or publication bias. Following the abstract and full-text screening, articles not evaluating the experiences of patients with lumbar radiculopathy symptoms and/or physiotherapy treatment were excluded.

Quality appraisal

The methodological strengths and limitations of the studies included in this research were assessed using the Critical Appraisal Skills Program (CASP) qualitative studies checklist [35,36]. This tool was chosen as it is considered the most effective for evaluating the quality of health-related qualitative studies and is endorsed by the Cochrane Qualitative and Implementation Methods Group's guidelines. Comprising 10 questions focusing on various methodological aspects, the CASP checklist aids in evaluating research strengths and limitations and promotes transparency, particularly beneficial for novice researchers. A summary table was created, detailing all aspects relevant to each question in the CASP qualitative research checklist. Additionally, the methodological strengths and limitations of each study were summarized narratively. Title and abstracts identified through database searches were exported to the reference manager (RefWorks), with duplicates subsequently excluded. These titles and abstracts were screened against eligibility criteria. Full texts of selected studies were then screened again for eligibility and quality. CASP was used solely to assess confidence in each review finding, not as a basis for exclusion. This approach aimed to identify gaps and assess the quality of existing literature.

Data extraction

Key features of primary studies were extracted from papers using a predetermined table, including data on setting, sample size, demographics, data collection, and synthesis methods used in primary qualitative studies. Data related to patient's illnesses and treatment representations, including actual quotes from patients and authors' interpretations, were extracted from results, discussion, and conclusion sections of primary studies.

Data synthesis

The best-fit framework synthesis approach was selected for this study, applying the RETREAT (Review question - Epistemology - Time/Timescale - Resources - Expertise - Audience and Purpose - Type of Data) framework. RETREAT outlines seven key factors considered by researchers influencing their choice of synthesis method, evaluating existing QES methods against these factors (Table 3).

The article "Understanding How Patients With Lumbar Radiculopathy Make Sense of and Cope With Their Symptoms" was retracted in 2025. Reasons: lack of ethics approval or compliance; concerns about the citations; concerns about the welfare of human subjects.

**Table 3:** The RETREAT criteria The RETREAT criteria were applied to select the data synthesis approach for this review [35,36]. RETREAT: Review question - Epistemology - Time/Timescale - Resources - Expertise - Audience and Purpose - Type of Data.

Criteria	Description
Research question	To explore patients' sense-making of their lumbar radiculopathy symptoms and evaluate cognitive/affective and behavioral responses
Epistemology	Interpretative
Time	Limited time frame
Resources	Single author with the support of university resources and tutors
Expertise	Novice researcher using qualitative evidence synthesis method for the first time
Audience and purpose	Target audience includes academics and healthcare professionals
Type of data	Qualitative studies

Framework synthesis, a deductive approach, was chosen to synthesize data from primary qualitative studies. This method involves mapping data onto a pre-identified framework comprising themes, concepts, ideas, or theories relevant to the phenomenon of interest. Best-fit framework synthesis (BFFS), a modified version, allows testing, refining, and building upon the a priori framework. While primarily deductive, BFFS incorporates inductive thematic analysis for data that does not fit the initial framework, making it both positivist and interpretive.

The Common-Sense Model of Self-Regulation (CSM) was selected as the theoretical model for this study. CSM posits that sense-making arises from patients' illness representations, reflecting perceived illness severity and threat. Cognitive and emotional representations form key domains, with cognitive representations further divided into identity, timeline, cause, control, and consequence subdomains.

These domains and subdomains of illness representation, including treatment, served as the a priori framework for categorizing findings from included studies into themes using BFFS. This approach aimed to depict patients' cognitive and emotional representations of lumbar radiculopathy, derived from their knowledge and experiences, reflecting the sense-making process.

The initial stages involved familiarization and identification of a thematic framework. After an extensive literature review on the phenomenon under investigation and leveraging the author’s expertise, the CSM was selected as the theoretical framework for this study. All included studies were thoroughly reviewed, and notes were taken to become familiar with the data. Quotes and authors' interpretations were coded against the illness representation domains derived from the CSM model. Themes outside these domains/subdomains were noted, coded, and thematically analyzed as independent constructs. These additional constructs supplemented the CSM framework. Relationships between CSM domains (and subdomains) were explored to develop succinct statements reviewing the findings based on the coded data.

The article "Understanding How Patients With Lumbar Radiculopathy Make Sense of and Cope With Their Symptoms" was retracted in 2025. Reasons: lack of ethics approval or compliance; concerns about the citations; concerns about the welfare of human subjects.

Confidence in review findings

This study utilized the GRADE‐CERQual (Confidence in the Evidence from Reviews of Qualitative research) approach to assess the certainty of evidence for drawing conclusions. Confidence in each finding was evaluated based on four key components: methodological limitations of included studies, coherence of review findings, adequacy of data contributing to review findings, and relevance of included studies to the review question. Confidence in review findings was judged as high, moderate, low, or very low based on supporting evidence.

Ethical considerations

This study adhered to the ethical standards of Sheffield Hallam University. After searching databases following the PRISMA checklist (Table 4), a total of 759 studies were identified. An additional study by Lin et al. [37] was identified from the reference list of Long et al. [38]. After removing duplicates (n = 113), the titles and abstracts of the remaining 646 studies were screened. Studies not qualitatively analyzing the experiences of patients with lumbar radiculopathy were excluded (n = 628). Of the remaining studies (n = 18), one [39] was excluded as it predates 2005, and another [40] was excluded for not evaluating the experiences of patients with lumbar radiculopathy symptoms and/or physiotherapy treatment, rendering them ineligible. Thus, 16 studies were included in the review. This process is graphically represented in the PRISMA flow diagram in Figure 1.

**Table 4:** PRISMA checklist PRISMA: Preferred Reporting Items for Systematic Reviews and Meta-Analyses.

Section and topic	Item	checklist item	Location where the item is reported
Title	1	Identify the report as a systematic review.	4
Abstract			
Abstract	2	See the PRISMA 2020 for Abstracts checklist.	4
Introduction			
Rationale	3	Describe the rationale for the review in the context of existing knowledge.	5
Objectives	4	Provide an explicit statement of the objective(s) or question(s) the review addresses.	12
Methods			
Eligibility criteria	5	Specify the inclusion and exclusion criteria for the review and how studies were grouped for the syntheses.	15
Information sources	6	Specify all databases, registers, websites, organizations, reference lists, and other sources searched or consulted to identify studies. Specify the date when each source was last searched or consulted.	14
Search strategy	7	Present the full search strategies for all databases, registers, and websites, including any filters and limits used.	64-67
Selection process	8	Specify the methods used to decide whether a study met the inclusion criteria of the review, including how many reviewers screened each record and each report was retrieved, whether they worked independently, and if applicable, details of automation tools used in the process.	15
Data collection process	9	Specify the methods used to collect data from reports, including how many reviewers collected data from each report, whether they worked independently, any processes for obtaining or confirming data from study investigators, and if applicable, details of automation tools used in the process.	17
Data items	10a	List and define all outcomes for which data were sought. Specify whether all results that were compatible with each outcome domain in each study were sought (e.g., for all measures, time points, analyses), and if not, the methods used to decide which results to collect.	15
	10b	List and define all other variables for which data were sought (e.g., participant and intervention characteristics, funding sources). Describe any assumptions made about any missing or unclear information.	15
Study risk of bias assessment	11	Specify the methods used to assess the risk of bias in the included studies, including details of the tool(s) used, how many reviewers assessed each study, whether they worked independently, and if applicable, details of automation tools used in the process.	16
Effect measures	12	Specify for each outcome the effect measure(s) (e.g., risk ratio, mean difference) used in the synthesis or presentation of results.	-
Synthesis methods	13a	Describe the processes used to decide which studies were eligible for each synthesis (e.g., tabulating the study intervention characteristics and comparing against the planned groups for each synthesis [item #5]).	15
	13b	Describe any methods required to prepare the data for presentation or synthesis, such as handling of missing summary statistics, or data conversions.	18-21
	13c	Describe any methods used to tabulate or visually display the results of individual studies and syntheses.	-
	13d	Describe any methods used to synthesize results and provide a rationale for the choice(s). If meta-analysis was performed, describe the model(s), method(s) to identify the presence and extent of statistical heterogeneity, and software package(s) used.	18
	13e	Describe any methods used to explore possible causes of heterogeneity among study results (e.g., subgroup analysis, meta-regression).	-
	13f	Describe any sensitivity analyses conducted to assess the robustness of the synthesized results.	-
Reporting bias assessment	14	Describe any methods used to assess the risk of bias due to missing results in a synthesis (arising from reporting biases).	21
Certainty assessment	15	Describe any methods used to assess certainty (or confidence) in the body of evidence for an outcome.	21
Results			
Study selection	16a	Describe the results of the search and selection process, from the number of records identified in the search to the number of studies included in the review, ideally using a flow diagram.	18
	16b	Cite studies that might appear to meet the inclusion criteria, but which were excluded, and explain why they were excluded.	18
Study characteristics	17	Cite each included study and present its characteristics.	20
Risk of bias in studies	18	Present assessments of risk of bias for each included study.	-
Results of individual studies	19	For all outcomes, present, for each study: (a) summary statistics for each group (where appropriate) and (b) an effect estimate and its precision (e.g., confidence/credible interval), ideally using structured tables or plots.	-
Results of syntheses	20a	For each synthesis, briefly summarize the characteristics and risk of bias among contributing studies.	-
	20b	Present results of all statistical syntheses conducted. If meta-analysis was done, present for each the summary estimate and its precision (e.g., confidence/credible interval) and measures of statistical heterogeneity. If comparing groups, describe the direction of the effect.	22-36
	20c	Present results of all investigations of possible causes of heterogeneity among study results.	-
	20d	Present results of all sensitivity analyses conducted to assess the robustness of the synthesized results.	-
Reporting biases	21	Present assessments of risk of bias due to missing results (arising from reporting biases) for each synthesis assessed.	-
Certainty of evidence	22	Present assessments of certainty (or confidence) in the body of evidence for each outcome assessed.	Appendix 5
Discussion			
Discussion	23a	Provide a general interpretation of the results in the context of other evidence.	32-37
	23b	Discuss any limitations of the evidence included in the review.	37,39,40,41
	23c	Discuss any limitations of the review processes used.	43
	23d	Discuss the implications of the results for practice, policy, and future research.	41-43
Other information			
Registration and protocol	24a	Provide registration information for the review, including the registered name and registration number, or state that the review was not registered.	-
	24b	Indicate where the review protocol can be accessed, or state that a protocol was not prepared.	-
	24c	Describe and explain any amendments to information provided at registration or in the protocol.	-
Support	25	Describe sources of financial or non-financial support for the review and the role of the funders or sponsors in the review.	-
Competing interests	26	Declare any competing interests of review authors.	-
Availability of data, code, and other materials	27	Report which of the following are publicly available and where they can be found: template data collection forms, data extracted from included studies, data used for all analyses, analytic code, and any other materials used in the review.	-

The article "Understanding How Patients With Lumbar Radiculopathy Make Sense of and Cope With Their Symptoms" was retracted in 2025. Reasons: lack of ethics approval or compliance; concerns about the citations; concerns about the welfare of human subjects.

**Figure 1:** PRISMA flow chart PRISMA: Preferred Reporting Items for Systematic Reviews and Meta-Analyses.

Description of studies

In adherence to the inclusion criteria, participants in the studies under review were individuals suffering from lumbar radiculopathy, either in acute or chronic form. The review encompasses studies documenting the experiences of patients exhibiting symptoms of lumbar radiculopathy [40-44] as well as those detailing their encounters with healthcare provision for the condition [8,45-49]. Notably, these studies exhibited no or very minor concerns regarding their quality, except for one study [50], which raised concerns about its rigor, and another [51], which questioned its reflexivity.

Framework synthesis

The data extracted from the studies were coded and aligned with the a priori domains and subdomains of the CSM. Initial themes and subthemes were derived through thematic analysis of the extracted data against these domains and subdomains. The need for additional inductive analysis was obviated by the sufficiency of the CSM in categorizing data related to sense-making. The raw data extracted from the included studies, along with the ensuing initial themes and subthemes, are visually represented in Table 5. Iterative identification of relationships among the extracted data culminated in the development of four overarching themes and their respective subthemes under the CSM domains of illness and treatment representations. Subsequently, the review findings were articulated.

**Table 5:** Concept table (key concepts)

Concept 1	Concept 2	Concept 3	Concept 4
Qualitative data extraction methods	Interview	Experiences	Lumbar radiculopathy
Patient beliefs	Focus groups	Views	Sciatica
Qualitative research	Case study	Perceptions	Sciatic neuropathy
Possible search terms	Open-ended questions	Opinions	Intervertebral disc displacement
		Knowledge	Nerve compression syndromes
		Attitudes	Radicular pain
		Feelings	Leg pain
		Beliefs	
		Sense	
		Sense-making	
		Meaning	
		Qualitative study	
		Qualitative methods	
		Qualitative research	

Table 6 presents the CSM DOMAIN of illness representations.

The article "Understanding How Patients With Lumbar Radiculopathy Make Sense of and Cope With Their Symptoms" was retracted in 2025. Reasons: lack of ethics approval or compliance; concerns about the citations; concerns about the welfare of human subjects.

**Table 6:** Overview of included studies RCT: Randomized controlled trial; PT: Physical therapy; SMT: Spinal manipulative therapy; HEA: Home exercise with advice.

Study	Duration of pain	Setting	Sampling method	Participants	Data collection	Data analysis	Quality
Pelletier et al., 2019 [48]	Chronic	Physiotherapy, nested in controlled trial, UK	Invites participants in the PT intervention arm of the RCT	21 participants opted in and out for surgery, 2 weeks after PT	Interview	Thematic analysis	No or very minor concerns
Goldsmith et al., 2019 [49]	Symptoms for >4 weeks	Musculoskeletal triage service	Consecutively sampled	13 English-speaking participants with unilateral radicular pain and no cauda equina symptoms	One-to-one interviews	Framework analysis	Minor concerns
Hofstede et al., 2013 [50]	Diagnosed within the previous two years	Leiden University Medical Center	Recruited via advertisements	≥18 years in 3 groups: Group 1 had symptoms, Group 2 conservative Rx, Group 3 waiting to decide on Rx	Interview in 3 focus groups	Thematic content analysis	No or very minor concerns
Maiers et al., 2016 [51]	Chronic	Alongside controlled trial, USA	Purposive sample nested within an RCT study	Volunteers for an RCT of 12 weeks of SMT, and SMT and HEA	Semistructured interview	Thematic content analysis	Minor concerns
Pollock et al., 2011 [52]	Mixed	General practice, combined with quantitative study, UK	Purposive sample nested within a large cohort study	Sciatica sufferers	Interviews (not specified)	Constant comparative method	Minor concerns
Reddington et al., 2021 [53]	Mixed	NHS primary healthcare sector, UK	Purposive sampling	33 English-speaking participants with a clinical diagnosis of sciatica	Thematic analysis	No or very minor concerns	
Ryan and Roberts 2018 [54]	Mixed	NHS primary healthcare sector, UK	Purposive sampling	14 participants of ≥18 years who recently underwent investigations for radiculopathy	Interview	Interpretative phenomenological analysis	No or very minor concerns
Ryan and Roberts 2019 [55]	3 months to 9 years	NHS, Musculoskeletal service in the UK	Purposive sampling	14 participants aged 34–81 years with a clinical diagnosis of sciatica	Interview	Interpretative phenomenological analysis	No or very minor concerns
Saunders et al., 2020 [56]	Approximately 7 months	General practices, NHS-based spinal clinics, and secondary care NHS trusts	Purposive sample nested within an RCT study	20 participants in the “fast-track” pathway, average age: 52 years	Interviews conducted at participants' homes, at the university, or via telephone	Framework analysis	No or very minor concerns
Rehman et al., 2019 [57]	At least 2 months	Neurosurgical practices	Convenient sampling	12 patients scheduled for surgical decompression for symptoms of sciatica	Semistructured interviews with patients and surgeons	Inductive content analysis	No or very minor concerns
van Dijk et al., 2022 [58]	Less than 6 weeks	Various healthcare settings (primary or secondary)	Convenient sampling	10 patients with actual or recent experience of sciatica, aged 30-70 years	In-depth semistructured interviews	Thematic analysis	Minor concerns
Svensson et al., 2013 [59]	3 years after treatment	Sahlgrenska University Hospital	Convenience sampling	20 patients treated by surgery and structured physiotherapy, aged 25–66 years	Interview guide with open-ended questions	Thematic analysis	No or very minor concerns

Theme 1: the overall illness experience

Finding 1: Overwhelming Experience With Neuropathic Pain

Studies noted that symptoms of radiculopathy, including neurological signs like dermatomal distribution of pins and needles, numbness, and myotomal distribution of weakness, proved more bewildering and debilitating than the pain itself [52-57]. Spontaneous pain was described as severe and incapacitating, with one participant likening it to "someone setting off a bomb" [53]. This was corroborated by participants reporting excruciating pain experiences [52].

The article "Understanding How Patients With Lumbar Radiculopathy Make Sense of and Cope With Their Symptoms" was retracted in 2025. Reasons: lack of ethics approval or compliance; concerns about the citations; concerns about the welfare of human subjects.

Finding 2: Difficulty in Understanding the Cause and Fear of Indications of a Serious Cause

Patients described the cause of lumbar radiculopathy as being "out of place" or "swollen," leading to "trapping" or "rubbing" of sensitive neural tissue [52-64]. Uncertainty regarding the triggering event and a lack of explanation from healthcare providers fueled fears of serious pathology [60-63].

Finding 3: Functional/Social/Recreational Limitations Due to the Impact of Lumbar Radiculopathy

Patients experienced disruptions in daily life, reduced physical strength, increased dependency, and difficulty in performing activities of daily living and leisure activities [6,65-67]. Work absenteeism, financial strain, disturbed sleep, and reduced social engagement were also reported [61].

Finding 4: Negative Emotional Response to the Impact of Lumbar Radiculopathy Which Increased With the Increased Duration of the Symptoms

All studies reported psychological distress among patients [6,52-67]. The inability to cope with symptoms, compounded by fear and dependency, led to heightened emotional distress, impacting the quality of life and relationships [6,52-67].

Discussion

The themes derived from the conceptual model elucidate how patients' beliefs and experiences with lumbar radiculopathy shape their illness and treatment representations. The discussion will explore how these representations influence coping strategies/behaviors and potential implications for clinical practice in addressing them effectively.

The article "Understanding How Patients With Lumbar Radiculopathy Make Sense of and Cope With Their Symptoms" was retracted in 2025. Reasons: lack of ethics approval or compliance; concerns about the citations; concerns about the welfare of human subjects.

Difficulty in Legitimizing Symptoms of Lumbar Radiculopathy

Patients struggled to cope with symptoms and articulate their experiences, amplifying frustration and stress. Uncertainty about the cause and prolonged symptoms hindered functioning and work, prompting information-seeking behaviors to validate symptoms and facilitate coping. The lack of credible information and healthcare provider explanations fueled fears of serious pathology, exacerbating anxiety and depression [68,69].

Comparison With the Literature

While diagnostic imaging can confirm pathology, it may also exacerbate fear and avoidance behaviors, leading to chronicity [68]. Addressing patients' concerns and providing reassurance and education about pain mechanisms can mitigate maladaptive behaviors and improve outcomes [70,71]. Efforts to improve self-efficacy through patient education, counseling, and promoting active coping strategies are crucial for long-term management [70-73].

Implications for Practice and Research

Strategies targeting illness representations through patient-centered approaches, psycho-education, and motivational interviewing can facilitate behavior change and improve outcomes [74-76]. Physiotherapists play a pivotal role in understanding patients' representations and addressing their informational needs to foster realistic understanding and coping. Education about pain mechanisms and self-management strategies can empower patients and enhance treatment adherence [77].

Future research should explore the impact of pain neuroscience education on illness representations and coping behaviors in patients with lumbar radiculopathy, employing qualitative methods to capture patient experiences and outcomes comprehensively.

Strengths and Limitations of the Study

This systematic review is the first to explore lumbar radiculopathy experiences through the lens of the CSM, providing insights into sense-making and coping behaviors. While the framework synthesis approach ensured rigor, limitations include the sole researcher conducting the study and potential biases. Future research should address these limitations and further explore the implications of illness representations on coping and treatment outcomes.

## Conclusions

Understanding how patients make sense of and cope with their symptoms of lumbar radiculopathy is essential for physiotherapists to anticipate and address coping behaviors, thereby influencing outcomes. Treatment strategies targeting illness representation can enhance patients' understanding of their symptoms and empower them to exert control over their condition through increased self-efficacy. The implications of employing the CSM in practice and guiding future research were identified in this study.

The article "Understanding How Patients With Lumbar Radiculopathy Make Sense of and Cope With Their Symptoms" was retracted in 2025. Reasons: lack of ethics approval or compliance; concerns about the citations; concerns about the welfare of human subjects.

## Appendices

**Table 7:** Raw data CSM: Common-Sense Model of Self-Regulation.

CSM domains/subdomains	Overarching themes	Subthemes	Data extracted
Cognitive representation			
Identity	Illness experience	Experience with symptoms	“Patients started with an enormous amount of pain, most often in their leg, and most often occurring spontaneously” [58]. “Altered sensations and weakness were perceived to be unpleasant, and to adversely affect balance and confidence in walking” [55]. “Pain like someone setting off a bomb” [52]. “can’t describe it… (it is) constant” [56] “... it was absolutely excruciating. I felt like ten knives were being rammed into my body. It was horrendous. It took me completely by surprise [55]. “It felt like someone had taken a knife and cut around the top of my leg and was peeling my skin down like you take off a stocking it was burning all the way down” [59].
		Difficulty in legitimizing their symptoms	“I feel like people have got no understanding of just how painful it can be. I don’t think it’s taken seriously enough. I don’t think people release just how painful it is. It is excruciating pain, constant” [59]. “I just wanted to be heard, wanted them to actually listen … I feel like people with sciatica pains they are branded with the same stick…I'm sure the person next door with sciatica … would be given the exact kind of thing to do [55].” “When I think about my leg I can feel the pins and needles going down it and the pain, I'm sure it's all in the mind” [56].
Cause	Concept of sciatica	Possible biomedical cause	…being “out of place” or “swollen”, causing either “trapping” or “rubbing” of sensitive neural tissue [56].
		Difficulty in understanding the cause	“I can't understand what triggered it off” [56]. “Your brain just ticks over and you think there could be some growth there … it's so severe and it's so constant” [58]. “I was like ‘Why can't I get up from my seat? Why are my legs not working? Am I paralysed?’” [57].
	Information-seeking behavior and the need for a diagnostic investigation to explain the cause of their symptoms	To facilitate coping	“I got a lot of the information from the internet, now I’m rubbish on the internet, somebody else got it for me…people who’ve had it, and what they’ve had done, and it’s got feedback and everything else [55].” “In six years I've never demanded an MRI. And I … called [her] bluff and even threatened … she said 'Okay, I'll send you for an MRI [54].” “Frustrated by the vagueness of their clinical diagnosis, participants wanted investigations to legitimise their symptoms, establish the cause, and to gain an accurate, definitive diagnosis. They thought that this information would help them to cope with symptoms and end rumination about a serious cause” [56]. “I was happy when I had the MRI because I knew what it was [causing the pain]; I think that’s half the problem because you worry about it otherwise … But he [the spinal specialist physiotherapist] showed me the MRI scan and showed me exactly where the disc bulge … I know what I’m coping with and I just feel easier now. That’s 90% of the battle really, that I know that it’s nothing too sinister [57]”. “So I say, dear neurologist, that’s not my spine. That’s a model on a table, my spine is in my back. And you think you can see on that model what’s wrong with my back? I thought I came here for a scan and to find out what’s in my back. No, he says, that MRI is only needed for the specialist pain team” [58].
		To facilitate treatment-related decision-making	“Receiving investigation results acted as a ‘turning point’ in management, enabling decisive treatment decision-making, and, for some, access to new options such as a consultant opinion” [59]. “For patients, the symptoms occurring from the bulge were the reason to seek medical aid” [59].
		When MRI fails to determine a cause	“When investigations failed to identify relevant findings, participants were unable to make sense of their symptoms, to relinquish the search for the cause, or to move forward in their management” [58].
Timeline	Consequences of the uncertainty of the duration of symptoms	Difficulty in coping due to shorter expected duration	“…their (patient’s) view of sciatica as resulting from a temporary and fixable ‘injury’ appears to have become an ongoing narrative, ingrained over time; despite this being contrary to their experiences of long-term symptoms. This sustained narrative of the temporariness of pain appears key to their lack of acceptance of pain as part of life, underpinning the biographical suspension experienced, and in turn leading to considerable frustration” [58] “The uncertainty of not knowing how long complaints would last and having no idea of the timeline was very difficult to cope with patients. Not only for their own well-being but also in relation to family and work demands” [57]. “(it) can be very tough… if you can't see any light at the end of the tunnel” [58]. If you said to me … there's a tablet, take that, you won't be in any pain tomorrow but you won't wake up, I think I would take it because I've had enough” [58].
		Effects on return to work	“…at its worst, it resulted in me taking three weeks off work, sick” [58]. “I've got to get back to work, for everybody … I'm just hoping to God this nerve block [injection] works. It's all fingers crossed, hold breath and just hope. I'm praying it works. If it doesn't, I don't know what I'm going to do” [58]. “Managing pain that was as long-lasting as sciatica meant that some people had to take regular time off work” [57]. “The pain and being unable to work, both. I have three months, that depends on how you are insured [as a freelancer], but I have to pay the first three months myself. So you want to get back to work as soon as possible” [58]. “I thought ‘well, okay, yes you can look at it that way as well’. I will just call my work: guys, I’m not doing well, you will see me in about three months, or something. So, um, well, that was a severe disappointment, as you can imagine” [58].
Consequences	Functional/social/recreational impact of pain		“My partner … needs to help me out of bed, get me to the bathroom … I couldn't put washing in … get the children dressed” [57]. “It started to affect my mobility, meaning that I couldn’t bend as much. I certainly couldn’t touch my toes anymore, which therefore meant I couldn’t put my knickers on in the morning properly, or put my socks on”[58]. “I had to cut down on all my fitness. I couldn’t go running. I had to stop playing football. I was in a lot of agony; it restricted me running round with the kids in the garden” [57]. “couldn't get into a comfortable position” [57]. “I feel as if I take my legs for a walk—not that they take me” [57]. “being left out of the loop” [58]”. “I like music … and there was the bike, and I love cooking …. I did none of those things I didn't go out for a walk, didn't go out for a meal, didn't go out to see anyone … for that period of time, life went on hold” [58].
	Effects on work		“I've never been unemployed. I've always worked and up until the last three years I was perfectly fit and healthy … seeing my life deteriorate … has been soul-destroying” [57].
Control	Difficulty in coping	Inability to cope	“I can cope with back pain. It’s the legs and the nerves and the bowels and the bladder that I find that scary, it is scary” [59].
		Reduced treatment adherence and self-management efficacy	“It reduces me to tears and at times and I can’t cope with that in my own mind somehow. I feel like I’m letting myself down by allowing it to take over” [57]. “I didn't want to feel a failure … I'm trying so hard to help myself, but it [exercise programme] was making it worse” [58].
	Coping strategies	Physical activity to avoid further disability	“She was afraid that she would not be able to walk at all in the future, and thus put a lot of energy into maintaining her mobility” [58]. “I am trying to do more … I'll leave here and I'll walk, probably three bus stops down… if I don't do that I'm not helping myself” [58]. “I’ve looked into Pilates classes as well … try and do anything that’s going to ease it or help” [58].
		Avoidance/restrictive strategies	“…sitting in a chair, trying to get comfortable and then, as soon as I was standing up, I get this shooting pain down my leg and I try to get the weight off my leg to try and stop the pain from going down my leg, and then eventually, you know, I do get a bit more mobile and then it’d go away”[56]. “I have come to terms with it now that I've just got to live with it, no one can do anything for me. That's what it is, that's what I do, struggle through. The days go on and that's it … I just be careful what I'm doing and restrict myself. I'd love to be able to go and do what I used to do in the garden and things. You've gone from an active person to … I don't know what” [53]. “I'd rather sit … in the corner than chat to people … a few years ago I'd have been… dancing” [53]. “… I just be careful what I'm doing and restrict myself. I'd love to be able to go and do what I used to do in the garden and things. You've gone from an active person to … I don't know what” [53]. “It was in the mental state where I was really frightened to leave the house, I thought that it was quite terrible that I didn’t dare go out of the house” [58]. “If I was lifting a lot and felt that I it was straining my back or something then I would stop immediately” [58]. “You can say that there are great limitations in what I can do, and that also makes me psychologically feel really bad” [58].
		Use of medication/drugs	“All you can do is lie there basically. Take a lot of painkillers” [57]. “I was having to do that (heroin) three or four times a week completely hammered because that’s the only way I could sleep” [58]. “It is a mixed feeling, I would prefer to quit all medication. I would prefer to, but I also notice that the medication is necessary to be able to move. That’s a very strange balance. It don't think it’s right, I struggle with it. Because I feel as if I do not function as the real me” [58].
Emotional representation	Negative emotional responses	Resignation to low mood frustration and anxiety	‘They also described becoming low in mood, anxious and having little tolerance for themselves” [58]. “My husband was really worried about me because one day it was particularly bad it was painful all day and by seven or eight in the evening, I was just grey and exhausted and miserable and crying” [57]. “It made me quite down and tearful, just mentally it took away my independence really. You are anxious, you are down. You take it out on people” [56].
		Suicidal thought	“[…] it’s like I’m constantly in excruciating pain. The idea of living to old age in this level of pain almost feels like it’s not an option. I’ve had, I guess you could consider, suicidal thoughts” [56]. “For others, the future held little hope and, for three of the fourteen participants, this had resulted in thoughts of suicide” [56].
		Changes from prior self	“I have come to terms with it now that I've just got to live with it, no one can do anything for me”[55]. “There's things I'm wary about now. Life has changed. Before I'd just pick something up, now I've got to be mindful how I'm bending over, how I'm turning. I'm fearful of it going again. Your life as you used to know it ain't the same, because your mind is mindful what could happen. You're always thinking about it. Always” [55].
Treatment representation			
Identity	Patient’s expectations from treatment	Reduce pain and increase mobility	“Well I’m hoping that it’ll help and I’ll be back on track back to normal I can’t see any reason for that not happening” [56]. “I hope that I’ll get some guidance on what is causing it and what to do to avoid it and hopefully to get back on my feet as soon as possible” [55]. “My thoughts were that it would assist my movement; I thought it would ease the pain a fair bit and also possibly relieve it enough so that I didn’t need to have surgery” [54].
		Prevent intake of medication and surgery	“So, I knew that at this point the drugs are just controlling the symptoms, they weren’t fixing the problems. Movement, exercise, and physio were going to be the thing that would fix the problem” [55]. “… also possibly relieve it enough so that I didn’t need to have surgery” [54]. “I think that it kind of gets you going in the morning and it just is good for your back. It's good for you. And if I hadn't come here, I wouldn't have been doing them” [56].
		Have no or opposite effect	“Well, I had had physio a couple of years ago in (place) and it was a total waste of time, a waste of time” [57]. “I should imagine a lot of exercises … would be unsafe. You’re in danger of making things worse. I wouldn’t want to push that disc any further than it is…” [54]. “I’m a bit wary about doing them now because of what they’ve told me about the bowel and bladder nerves” [56].
Timeline	Accelerated access to physiotherapy reduced the physiological and psychological impact		“I think it was absolutely essential to me to be seen quickly. The effect it has physically is terrible but the effect on my mental health was even worse. Having to wait another 6 weeks would have been bad for me physically. But mentally it would have devastated me” [54].
Consequence (treatment effect – including advice)	Reduced pain and increased mobility		“[the physiotherapy helped to keep] the flexibility and my body supple so that as soon as I’d had my surgery, my body was ready to do the exercises” [57]. “The ability to perform exercises which relieved pain, improved movement and were confidence building was especially welcomed” [58]. “The flexing of the spine and the stretching of the spine were the two things that really got me loosened up and made me feel like I could stoop over, walk normal, not drag my one leg” [57].
	Improved exercise adherence		“It has made me start exercising, which is probably a good thing. The physio has got me into doing exercises on a daily basis” [53]. “the commitment that, yep, that's a daily thing that's going to be done” [54]. “The advice was really useful I think in the first instance, knowing that it was safe to go swimming for instance is what I needed really because I didn’t really know” [57].
	Preference for individualized treatment		“Patients recounted the effectiveness of giving them the time and opportunity to relate their experience, combined with a full clinical explanation in helping them cope with their sciatica” [57]. “…they mentioned that some professionals had a lack of attention for their anxiety, personal situation, and preferences, while the elicitation of patient preferences is crucial to SDM” [53]. “Those who responded positively appreciated the way it was tailored to their individual condition” [57]. “The aspect of the intervention which participants in both groups found most useful was the clarity of individualized advice and education about sciatica” [56].
Control	Treatment and education aiding self-management	Increased physical activity and exercise adherence	“I’m no longer in fear of the fact that if I do something like pick something up or bend over, I’ve no fear because in my head it would all go wrong from there, that has been taken away from me which is very very useful” [59]. “…really opened my eyes on how much more activity I could do under the circumstances that I'm in…I didn't have any clue that I could be that active, and that I should be active” [59]. “… have become an issue of strengthening and getting more movement back rather than managing pain, the original reason for coming. Real shifting goals” [59]. “Some patients said that when symptoms arose they were often able to deduce why, which made it easier to cope with their symptoms. Others reported that they were sometimes able to decrease symptoms when they arose. Patients also expressed that they tended not to avoid doing things, but instead reflected and worked out new ways to perform the activity” [59].
	A desire for credible information		“I took into account mainly the information that was given to me … specifically the back pain … the origin and how I could reduce it. What kinds of things could I do for the long term? I think that's what probably what interested me the most” [51]. “The importance of clear information and explanation emerged from many of the accounts, and they felt that this would help them cope with the diagnosis and prognosis” [52]. “…timely, clear and understandable advice and education was important to most participants” [53].
Post-treatment emotional representations	Promoted emotional well-being	Increased confidence and reduced avoidance	“A lot of it was the confidence side of things and the counseling that I got from the physiotherapist that you can bend like this and pick up something quite heavy and also the development of the exercises to get over the psychological side of thing” [48]. “I’m no longer in fear of the fact that if I do something like pick something up or bend over, I’ve no fear because in my head it would all go wrong from there, that has been taken away from me which is very very useful” [53].
		Helped in legitimizing symptoms	“It's more a personal emotional thing than a physical thing, it was again that [provider] was so extremely attending to me. He was always, really trying to see the person in me, and work with that, and seek out things. This was what I enjoyed most that I was taken so seriously…” [51]. “It was excellent, so good I can’t tell you. I felt that (physiotherapist) had time for me, he supported me mentally, he cared and listened and supported me to improve both mentally and physically.” [53] “I felt that I was respected as an individual, I felt like she had time to listen to me and was obviously a specialist in her field and definitely knew what she was talking about” [53].
		Improved mood	“It's added more quality to my life…I'm even happier!” [51]. “It gave me back a normal life. When you're in pain so much of the time…your whole outlook is down. It's like I have a new outlook on life now” [51].

The article "Understanding How Patients With Lumbar Radiculopathy Make Sense of and Cope With Their Symptoms" was retracted in 2025. Reasons: lack of ethics approval or compliance; concerns about the citations; concerns about the welfare of human subjects.

**Table 8:** Confidence in review findings CSM: Common-Sense Model of Self-Regulation; CERQual: Confidence in the Evidence from Reviews of Qualitative research.

Finding	Review Findings according to CSM	Methodological Limitation	CERQual Confidence Assessment
Overwhelming experience with neuropathic pain	Saunders et al., 2018 [56]; Saunders et al., 2020 [65]; Ryan and Roberts 2019 [54]; Pollock et al., 2020 [52]; Goldsmith et al., 2019 [49]; Hofstede et al., 2013 [50]; van Dijk et al., 2022 [58]; Maiers et al., 2016 [51]; Pelletier et al., 2015 [48]; Reddington et al., 2021 [53]; Svensson et al., 2013 [59]; Rehman et al., 2019 [57]	Minor concerns due to the unclear rigor and the reflexivity of the studies Goldsmith et al., 2019 [49] and Pollock et al., 2020 [52]	None or very minor concerns. The cogency of the finding was well supported by the data in the underlying studies.
Difficulty in understanding the cause and fear of indications of a serious cause	Goldsmith et al., 2019 [49]; Reddington et al., 2021 [53]; Ryan and Roberts 2019 [54]; Ryan and Roberts 2018 [55]; Pollock et al., 2020 [52]	Minor concerns due to the unclear rigor and the reflexivity of the studies, Goldsmith et al., 2019 [49] and Pollock et al., 2020 [52]	None or very minor concerns. The cogency of the finding was well supported by the data in the underlying studies.
Functional/social/recreational limitations due to the impact of lumbar radiculopathy	Ryan and Roberts 2018 [55]; Pelletier et al., 2015 [48]; Pollock et al., 2020 [52]; Saunders et al., 2018 [56]; Svensson et al., 2013 [59]	Minor concerns due to the unclear rigor of the study Pollock et al., 2020 [52]	None or very minor concerns. The cogency of the finding was well supported by the data in the underlying studies.
Negative emotional response to the impact of lumbar radiculopathy which increased with the increased duration of the symptoms	Saunders et al., 2018 [56]; Ryan and Roberts 2019 [54]; Pollock et al., 2020 [52]; Goldsmith et al., 2019 [49]; Hofstede et al., 2013 [50]; van Dijk et al., 2022 [58]; Maiers et al., 2016 [51]; Pelletier et al., 2015 [48]; Reddington et al., 2021 [53]; Rehman et al., 2019 [57]; Svensson et al., 2013 [59]	Minor concerns due to the unclear rigor and the reflexivity of the studies Goldsmith et al., 2019 [49] and Pollock et al., 2020 [52]	None or very minor concerns. The cogency of the finding was well supported by the data in the underlying studies.
Physical activity to avoid further worsening of the consequences	Pollock et al., 2020 [52]; Ryan and Roberts 2019 [54]	Minor concerns due to the unclear rigor and the reflexivity of Pollock et al., 2020 [52]	None or very minor concerns. The cogency of the finding was well supported by the data in the underlying studies.
Avoidance/restrictive behaviour to avoid the pain experience and emotional consequences	Pollock et al., 2020 [52]; Ryan and Roberts 2019 [54]; Sauders et al., 2018 [56]; Reddington et al., 2021 [53]; Svensson et al., 2013 [59]	Minor concerns due to the unclear rigor and the reflexivity of Pollock et al., 2020 [52]	None or very minor concerns. The cogency of the finding was well supported by the data in the underlying studies.
Taking medications (not always preferred) or also drugs to cope	Pelletier et al., 2015 [48]; van Dijk et al., 2022 [58]; Reddington et al., 2021 [53]	Minor concerns due to the unclear rigor and the reflexivity of van Dijk et al., 2022 [58]	None or very minor concerns. The cogency of the finding was well supported by the data in the underlying studies.
Demonstration of information-seeking behavior	Ryan and Roberts, 2018 [55]; Svensson et al., 2018 [59]; Ryan et al., 2020 [62]; Ryan and Roberts, 2018 [55]	No concerns	None or very minor concerns. The cogency of the finding was well supported by the data in the underlying studies.
Expectations for exercise to reduce pain and increase mobility	Hofstede et al., 2013 [50]; Goldsmith et al., 2019 [49]; Reddington et al., 2022 [61]; Pelletier et al., 2015 [48]	Minor concerns due to the unclear rigor and the reflexivity of Goldsmith et al., 2019 [49]	None or very minor concerns. The cogency of the finding was well supported by the data in the underlying studies.
Expectations for exercise to reduce intake of medication and prevent surgery	Reddington et al., 2021 [53]; Pelletier et al., 2015 [48]	No concerns	None or very minor concerns. The cogency of the finding was well supported by the data in the underlying studies.
Expectations for exercise to have no or opposite effect (worsen the condition)	Reddington et al., 2022 [60]; Goldsmith et al., 2019 [49]	Minor concerns due to the unclear rigor and the reflexivity of Goldsmith et al., 2019 [49]	None or very minor concerns. The cogency of the finding was well supported by the data in the underlying studies.
Benefits of accelerated access to treatment	Reddington et al., 2022 [60]; Ryan et al., 2020 [62]	No concerns	None or very minor concerns. The cogency of the finding was well supported by the data in the underlying studies.
Treatment helped to reduce pain and increase mobility as expected	Pelletier et al., 2015 [48]; Maiers et al., 2016 [51]; Reddington et al., 2022 [60]; Saunders et al., 2018 [56]	No concerns	None or very minor concerns. The cogency of the finding was well supported by the data in the underlying studies.
Treatment and education improved exercise adherence and self-efficacy aiding better self-management. Preference to individualized and patient-centred treatment and education	Maiers et al., 2016 [51]; Pelletier et al., 2015 [48]; Sauders et al., 2018 [56]; Reddington et al., 2022 [60]; Svensson et al., 2013 [59]	No concerns as studies done in 3 different countries	None or very minor concerns. The cogency of the finding was well supported by the data in the underlying studies.
